The article "Measuring and Modelling Nonlinear Elasticity of Ex Vivo Mouse Muscles" was published in 2021. Journal: J Healthc Eng.

# Measuring and Modelling Nonlinear Elasticity of Ex Vivo Mouse Muscles

**DOI:** 10.1155/2021/5579232

**Published:** 2021-11-17

**Authors:** E. Rizzuto, R. De Luca, A. Musarò, Z. Del Prete

**Affiliations:** ^1^Department of Mechanical and Aerospace Engineering, Sapienza University of Rome, Rome, Italy; ^2^Laboratory Affiliated to Istituto Pasteur Italia—Fondazione Cenci Bolognetti, DAHFMO-Unit of Histology and Medical Embryology, Sapienza University of Rome, Rome, Italy

## Abstract

Elastography is a noninvasive imaging technique that provides information on soft tissue stiffness. Young's modulus is typically used to characterize soft tissues' response to the applied force, as soft tissues are often considered linear elastic, isotropic, and quasi-incompressible materials. This approximation is reasonable for small strains, but soft tissues undergo large deformations also for small values of force and exhibit nonlinear elastic behavior. Outside the linear regime, the elastic modulus is dependent on the strain level and is different for any kind of tissue. The aim of this study was to characterize, ex vivo, the mechanical response of two different mice muscles to an external force. A system for transverse force-controlled uniaxial compression enabled obtaining the stress-strain (*σ*-*ε*) curve of the samples. The strain-dependent Young's modulus (SYM) model was adopted to reproduce muscle compression behavior and to predict the elastic modulus for large deformations. After that, a recursive linear model was employed to identify the initial linear region of the *σ*-*ε* curve. Results showed that both muscle types exhibited a strain hardening effect and that the SYM model provided good fitting of the entire *σ*-*ε* curves. The application of the recursive linear model allowed capturing the initial linear region in which the approximation of these tissues as linear elastic materials is reasonable. The residual analysis displayed that even if the SYM model better summarizes the muscle behavior on the entire region, the linear model is more precise when considering only the initial part of the *σ*-*ε* curve.

## 1. Introduction

Noninvasive measurement of soft biological tissues' mechanical properties is of significant clinical interest as pathologies are generally correlated with changes in tissue stiffness. Many cancers, such as breast and prostate ones, typically appear stiffer than the surrounding tissues, and diffuse diseases, such as cirrhosis of the liver, are known to significantly increase the stiffness of the liver tissue as a whole [1–5]. In addition to pathology, there is evidence that consistent elastic contrast also exists among various normal tissues [1, 6, 7]. Imaging these differences in soft tissue stiffness is commonly obtained using elastography [2, 3, 8–11], which provides noninvasive images of tissue mechanical characteristics, at depth, with high resolution and good contrast.

To date, there are several elastography imaging techniques which are based on the same principle: an external force is applied to the tissue, and the local internal displacement is measured by either ultrasound or magnetic resonance imaging to be converted in a suitable parameter to display (e.g., strain, Young's modulus, and shear wave speed). The external force may be applied in different ways: a dynamic force is mandatory to generate a shear wave and thus to measure and image its speed, while the applied force may be dynamic, quasistatic, or static if there is need to image displacement or strain [2, 3]. The importance of measuring tissue mechanical properties lies in the fact that they may be considered diagnostic indicators which provide additional and clinically relevant information for the characterization of soft tissues and for the discrimination between normal and abnormal tissues. In this context, a wide experience with transient and shear wave elastography to assess diffuse liver diseases exists [3, 9, 12]. Transient elastography allows for a reduction of more than 50% of liver biopsies which, to date, still represents the gold standard technique for the diagnosis of liver chronic disease, even if biopsies are invasive and painful and may cause anxiety to the patients [13, 14]. Strain and shear wave elastography are typically used to examine breast, thyroid, gastrointestinal tract, prostate, and musculoskeletal system [9, 15–18]. For instance, shear wave elastography improves the specificity of breast ultrasound imaging, has high reproducibility for breast masses [19–22], and provides information of the functional changes accompanying musculoskeletal pathologies [23–25].

Soft tissues are viscoelastic, poroelastic, anisotropic, and nonlinear materials. In practice, many assumptions are made to display their mechanical properties using elastography: they are typically modelled as linear elastic, isotropic, and quasi-incompressible materials [6]. Under these conditions, one single parameter is needed to characterize the response of a tissue to the applied mechanical force: Young's modulus [6, 26]. However, when scanning with the ultrasound probe, a precompression is applied by the operator, and soft tissues, being nonlinear, exhibit a strain hardening effect; that is, they get stiffer as the amount of applied pressure increases [27, 28]. For large deformations, they show a nonlinear elastic behavior as their modulus is dependent on the strain level, and the increase in the modulus varies from one tissue type to another [6, 29, 30]. In strain elastography, large strains may be required to achieve a reasonable strain signal-to-noise ratio and to enhance the contrast between healthy and pathological tissues [30]. Nevertheless, strains outside the linear elastic region do not provide reliable information about tissue material properties, since Young's modulus for high strain is largely stress-dependent [26]. High strain elasticity measurements provide information only about tissue pseudoelastic properties, that is, elasticity of tissue at a specific stress or strain level. In shear wave elastography, the probe must be applied very lightly with a generous amount of gel [25, 31]; otherwise, abnormal stiffness is shown; for instance, in breast imaging, fat tissue may be measured to have the same elasticity pattern of cancer if a high precompression is applied [29]. A proper assessment of the force applied during elastography techniques may be therefore used, together with the proper mathematical model, as a real-time correction of the measurements to avoid misinterpretation of the results.

Within this context, the present work aims at investigating and modelling the elastic behavior of two different mice muscles. A mechanical system able to apply an external force and to simultaneously measure the subsequent displacement of the sample is used to obtain, *ex vivo*, the stress-strain (*σ-ε*) curves of Tibialis Anterior (TA) and Extensor Digitorum Longus (EDL) muscles. These curves are then employed to find the mathematical models that describe the elastic behavior of the investigated soft tissues and to identify the limits of the linear stress-strain regions, as well as to reconstruct the Young's modulus values corresponding to high strain levels.

## 2. Theory

The elasticity of a solid material describes its tendency to return to the original shape and size after being subjected to a deforming force. Soft biological tissues are nonlinear, viscoelastic, anisotropic, and nonhomogeneous materials, and their properties are dependent on time. Moreover, the resistance to deformation increases when the applied stress increases [32], so that multiple values of Young's modulus could be obtained, as it depends on the applied stress [26, 32]. In general, it is assumed that soft biological tissues behave as linear elastic, isotropic materials [32] but, *in vivo*, soft tissues usually undergo large deformations and these assumptions become invalid [33]. To characterize the nonlinear elastic response of soft tissues and to overcome the difficulty in obtaining Young's modulus by force-deformation test, several theoretical models have been formulated [33, 34]. In particular, Li et al. [35] proposed a strain-dependent Young's modulus (SYM) to introduce nonlinearity in the general theory of elasticity for transversely isotropic bodies, as reported in the following equation:

(1) $$\begin{array}{c} E_{L}=k_{1}e^{k_{2}\varepsilon },\\ E_{T}=k_{3}e^{k_{4}\varepsilon }, \end{array}$$

where *E*_*L*_ and *E*_*T*_ are the longitudinal and transverse Young's moduli, respectively, and *k*_1_, *k*_2_, *k*_3_, and *k*_4_ are the model parameters. The authors applied this model to reproduce the tensile behavior of porcine aortic heart valves, whereas Van Loocke and coauthors [33, 36] adapted it to reproduce skeletal muscle tissue compression behavior. In our study, the SYM model was used to investigate the passive elastic behavior of *ex vivo* mouse skeletal muscles, and model parameters are determined by fitting the experimental data (*ε*, *σ*).

## 3. Experimental Setup and Protocol

### 3.1. Animals

Six C57BL/6 female mice (15–17 week old), bred at the DAHFMO-Unit of Histology and Medical Embryology Laboratories at Sapienza University of Rome, were used. All the experiments were conducted within the animal welfare regulations and guidelines of the Italian national law D.L. 04/03/2014, n.26, about the use of animals for research. From each animal, one Tibialis Anterior (TA) muscle and one Extensor Digitorum Longus (EDL) muscle were excised and subjected to uniaxial unconfined compression in the cross-fiber. After the dissection, the samples were kept soaked in a physiological solution at room temperature and the measurements were completed within 30 minutes. As the test typically lasted few minutes, dehydration of the sample was not an issue. No preconditioning was applied to the samples and each sample was tested once to avoid permanent deformation due to the high strain level induced [36]. A preload ranging from 6 mN to 9 mN was applied to the sample to attach it to the indentor.

### 3.2. Uniaxial Unconfined Compression Test

Two methods are typically employed to assess the mechanical characteristics of soft biological tissues: probe indentation and tensile stretching. Even though both techniques provide a description of the material response to an applied stress, they are distinct. Strictly speaking, the adopted method of deformation must be considered to make empirical values of Young's modulus reliable, consistent, and nonambiguous [32]. In this study, a force-controlled uniaxial compression test has been conducted on fresh mouse tissues *ex vivo* [37]. The experimental system was based on a dual mode actuator/transducer 305C-LR (Aurora Scientific Inc., Aurora, Canada) able to measure and control both length and force, with length signal resolution of 1 *μ*m and force signal resolution of 1 mN. The motor was controlled through a DAQ NI-PCIe-6363X (National Instruments, Austin, TX, USA), and custom-made software developed in LabView 2012 (National Instruments, Austin, TX, USA) allowed setting the shape and the intensity of the applied loading profile. A circular indentor (Aurora Scientific Inc., Aurora, Canada) of 3 mm of diameter was rigidly attached to the lever arm of the actuator/transducer. The sample was placed in touch with the piston with the muscle fibers perpendicular to the direction of compression and remained unconstrained laterally. The motor was controlled in force and the specimen was subjected to a compressive ramp whose maximum force was 200 mN at 50 s. The loading speed was set at 4 mN/s and was chosen reasonably low to limit the viscosity effects. The applied signals were force-controlled to mimic the use of a scanning probe in elastography applications, and the true applied force and displacement were recorded for offline processing. All the instrumentations were placed on an isolation workstation with Faraday cage (Newport Vision IsoStation, California, USA).

### 3.3. Recursive Linear Fitting Model

Even though soft biological tissues exhibit a nonlinear *σ-ε* behavior, they are typically assumed to be linear elastic if a significant linear region of the *σ*-*ε* curve exists in the limit of small deformation to the applied stress [32], and elastography is generally based on this approximation [3, 6, 26]. Here, a recursive linear fitting model was developed to calculate the strain range in which each tested sample could be reasonably considered a linear elastic solid. This model yielded to obtain the best linear fitting curve in terms of *R*^2^ value, thus allowing to assess the highest deformation (*ε*_max_) of the linear regime. Young's modulus of the linear region (*E*_lin_) was then obtained as the slope of this curve [37].

### 3.4. Optical System to Measure Sample Characteristic Dimension

Measurement of the sample geometrical dimensions was made using an optical methodology. This system consisted of an ACA2040-180 km monochromatic camera (Basler, Ahrensburg, Germany) mounted on a SMZ800N (Nikon Inc., Melville, NY, USA) stereomicroscopy equipped with a 0.5 Plan Apo objective (Nikon) to capture the whole longitudinal length of the specimen. This camera had a pixel size of 5.5 *μ*m × 5.5 *μ*m and a full resolution of 2048 × 2048 pixels. The lighting was provided by a PL-3000 cold light illuminator (Photonic Optics, Vienna, Austria) that guaranteed a light field intensity up to 26 Mlx, and a NI-PCIe 1433 frame grabber (National Instruments, Austin, TX, USA) was employed for image acquisition. A 45° angled mirror (Nikon) was used to image the transverse length *w*_0_ of the sample (Figure 1).

For each test, an image prior compression was acquired to assess the number of pixels (*N*_*p*_) in the length (*h*) of the circular piston (Figure 1(a)), which was used as calibrating target. Being *h* = 1.00 mm (this measurement was made using an analog caliper with an accuracy of 0.05 mm), the pixel size was obtained dividing *h* by *N*_*p*_. This value was then used to calculate the width (*w*_0_) of the specimen when the preload was applied (Figure 1(b)). All the pixel assessments were done by using ImageJ software (National Institutes of Health, Bethesda, Maryland, USA). The average characteristic dimension *w*_0_ of the specimens was 2.00 ± 0.28 mm and 0.89 ± 0.11 mm for the TA and EDL groups, respectively.

### 3.5. Statistical Analysis

Differences in the measured maximum strain, in the maximum value of Young's modulus computed with the SYM model, in the maximum strain value computed with the linear model, and in the maximum value of Young's modulus computed with the linear model between EDL and TA groups were evaluated with unpaired *t*-test, and the difference was considered significant for *p* value <0.05. Differences in the residual distributions between the linear model and the SYM model were evaluated with Mann–Whitney rank-sum test, and the difference in the median values between the two groups was considered significant for *p* value <0.05. Statistical analysis was performed with GraphPad Prism 6.0 (GraphPad Software, Inc).

## 4. Results and Discussion

Figure 2 shows the mean and standard deviation of the strain-stress relationship measured from the applied force and the consequent displacement of 5 TA muscles and 6 EDL muscles. As expected, for both muscle types, the strain increased nonlinearly as a function of the applied stress, and each muscle type exhibited a different elastic behavior. In particular, the average maximum strain value was 43% higher (*p* < 0.01) in the EDL group than in the TA group.

To quantify the strain hardening effect of the investigated mouse muscles, the exponential fitting proposed by Li et al. [35] was exploited. The adopted model provided a very good fit to the experimental data, as shown in Table 1, and allowed reconstructing the values of Young's modulus for each level of strain undertaken by each specimen.

Figure 3(a) shows an example of the experimental results fitted with the exponential model for a TA sample, and Figure 3(b) displays the corresponding reconstructed Young's modulus as a function of strain. Of note, the average maximum Young's modulus obtained from the SYM model was significantly (*p* < 0.01) higher in the TA muscles than in the EDL muscles.

Table 2 displays reconstructed *E*_lin_ and *ε*_max_ obtained through the recursive linear fitting for both muscle types. Results showed that the initial region of the *σ-ε* curve is highly linear (*R* > 0.98) for strains up to 8.18 ± 1.51%, on average, for TA muscles, and to 13.26 ± 2.29%, on average, for EDL muscles, with this difference being statistically significant (*p* < 0.01). As a result of this, Young's modulus associated with the entire linear region was found to be 38.12 ± 13.91 kPa, on average, for TA muscles, and 33.46 ± 6.5 kPa, on average, for EDL muscles. The higher variability obtained for the linear model is, in our opinion, related to the fact that this value is computed on the very first part of the stress-strain curve, the one with the higher slope. Any small differences in the maximum strain determined on the basis of our recursive algorithm may therefore lead to high differences in the *E* values. Nonetheless, this variability obtained in the estimated modulus even for samples that are excised from very similar and controlled animal confirms the need for assessing the exact elasticity for each sample of interest.

Figure 4 depicts an example of the two fitting models for one EDL specimen, highlighting that, for small strains, the linear model provides better fitting than the exponential one.

To evaluate the goodness of fitting, we performed a residual analysis for the two models: for each specimen, we focused on the initial linear region of the *σ*-*ε* curve previously computed and calculated the difference between the measured value and the value reconstructed with the linear model and with the SYM model, respectively.  Table 3 shows the results obtained for all the specimens, and Figure 5 shows an example of the results for one EDL muscle: for all the tested specimens, except for the initial and the final portion of the analyzed curve, in which the residuals are very similar for the two tested models, in the central part of the curve, the linear model better describes the experimental data. As a result of this, the average value of the linear model's residuals was lower than the average value of the SYM model's residual for all the tested specimens. When comparing the residual distributions, a statistically significant difference was found for all the tested specimens except that for one TA (Table 3), with the residuals computed for the linear model being extremely lower than residuals computed for the SYM model.

## 5. Conclusions

The aim of this study was to characterize, *ex vivo*, the mechanical response of two different types of mice muscles to an external force, the Tibialis Anterior (TA) and the Extensor Digitorum Longus (EDL), by introducing the nonlinearity in the general theory of linear elasticity. Elastography techniques are based on Hooke's law by assuming that soft tissues act as linear elastic materials; however, under large deformations, they exhibit a nonlinear elastic behavior, and a proper understanding of their mechanical properties is necessary to avoid errors in the elastogram and in the interpretation of the results. Indeed, the possibility of a more accurate identification of tissues' mechanical properties results indeed crucially in elastography approach. The comparison between the average strain values undergone by TA and EDL muscles showed that they exhibit distinct strain hardening effects, with the EDL being more compliant. The use of the SYM model already employed for the porcine hearth aortic valve [35] and to assess the passive behavior of skeletal muscle in compression [33, 36] provided a very good fit to the experimental data. The SYM model allowed to characterize how fast the stiffness of each specimen was raised with the increase of the applied load outside the linear elastic region and to predict Young's modulus for large deformations. Because of a more compliant behavior of EDL muscles, the maximum value of Young's modulus obtained through the SYM model resulted to be significantly higher in TA muscles. However, the SYM model did not allow getting a single *E* value to be associated with each muscle type. Due to the high variability of the strain as a function of the stress under large deformations, in strain elastography, reasonable strain signal-to-noise ratio and strain contrast between these two tissues may not be reached, and, in shear wave elastography, they may be measured having the same elasticity. The use of a recursive technique allowed obtaining an assessment of the part of the region in which the tissue linear response is more prevalent on the nonlinear one. Interestingly, even if the SYM model provided a good fitting of the entire *σ*-*ε* relationship, in the initial part of the curve, the linear model provided an even more accurate modelling. This linear region was found to reach a higher strain value, on average, for EDL muscles than for TA ones, in accordance with the more compliant behavior previously measured for EDL specimens. Once the linear region was identified, it was possible to associate a unique value of Young's modulus to each muscle type, reducing the likelihoods of misinterpretation of the elastography outcomes. Again, it has to be remarked that the high variability obtained in the estimated linear modulus even for samples that are excised from very similar and controlled animal confirms the need for assessing the exact elasticity for each sample of interest. Of note, in this study, the tissue viscosity was considered negligible, but biological tissues, being viscoelastic, exhibit a stress dependence on the rate of straining. Anyway, our specimens were tested at a very slow rate to perform quasistatic indentations, minimizing the effect of viscoelasticity. As expected, the strain as a function of the stress exhibits a high variability; therefore results from this experimental study encourage the adoption of the models employed here to predict both the nonlinear and linear elastic responses of compressed soft tissues to provide, together with the measurement of the force applied during elastography techniques, a real-time correction of the measurements to avoid misinterpretation of the results. Finally, an improved version of the model proposed here may be therefore developed to consider the small contribution of viscosity, which can also contribute to reducing the variability obtained for the linearized values of *E*.

## Figures and Tables

**Figure 1:** Example of images of a TA muscle acquired by the optical system. The indentor and the lever arm of the actuator/transducer were also captured. (a) Precompression image: *h* is the length of the circular piston. (b) Image acquired after a preload of 8 mN was applied: *w*_0_ is the initial length of the sample in the cross-fiber direction.

**Figure 2:** Mean (solid line) and standard deviation (dotted line) of the experimental strain-stress curve for the TA (grey) and EDL (black) groups of samples. Average data are expressed as mean ± SD. *n*: 5 TA and 6 EDL.

**Figure 3:** (a) Experimental stress-strain curve of one TA specimen (solid) and the corresponding exponential fitting model curve (dotted). (b) Reconstructed Young's modulus as a function of the strain level.

**Figure 4:** Example of fitting curves (dotted grey: SYM model; solid grey: linear model) and experimental data (black) for an EDL specimen.

**Figure 5:** Example of a residual analysis for an EDL specimen (*n*: 2 in Table 2) computed in the initial linear region for the two applied models (a) and their frequency distribution (b).

**Table 1:** *R* ^2^ values of exponential models and the corresponding maximum value of the reconstructed Young's modulus for TA and EDL specimens.

Mouse	TA		EDL	
	*R* ^2^	*E*_max_ (kPa)	*R* ^2^	*E*_max_ (kPa)
1	0.9992	138.65	0.9984	75.33
2	0.9996	130.34	0.9976	87.98
3	0.9994	121.69	0.9963	80.59
4	0.9994	118.62	0.9989	105.64
5	0.9974	101.61	0.9973	70.58
6	—	—	0.9987	97.06
Average		122.18 ± 13.91^*∗∗*^		86.20 ± 13.36

Data reported here refer to the whole loading profile. Average data are expressed as mean ± SD. ^*∗∗*^*p* < 0.01 versus EDL.

**Table 2:** *R* ^2^ values of the linear model for TA and EDL specimens in the initial region of the stress-strain curve.

Mouse	TA			EDL		
	*R* ^2^	*E*_lin_ (kPa)	*ε*_max_ (%)	*R* ^2^	*E*_lin_ (kPa)	*ε*_max_ (%)
1	0.9909	52.29	8.37	0.991	37.18	16.11
2	0.9897	56.73	7.05	0.9954	36.84	12.61
3	0.9878	29.56	8.61	0.9913	26.24	14.45
4	0.9866	25.71	6.52	0.9944	38.55	11.14
5	0.9813	29.29	10.39	0.9898	24.07	14.97
6	—	—	—	0.9855	37.89	10.28
Average		38.72 ± 14.58	8.18 ± 1.51^*∗∗*^		33.46 ± 6.50	13.26 ± 2.29

^*∗∗*^ *p* < 0.01 versus EDL.

**Table 3:** Residuals (Pa) of the linear model and the SYM model in the initial linear region of the stress-strain curve.

Mouse	TA		EDL	
	Linear model	SYM model	Linear model	SYM model
1	148.52 ± 87.21	243.35 ± 186.80^*∗∗*^	235.71 ± 122.02	323.63 ± 194.28^*∗∗*^
2	127.71 ± 71.76	182.12 ± 102.46^*∗∗∗*^	137.22 ± 86.71	437.38 ± 299.13^*∗∗∗∗*^
3	134.46 ± 79.46	194.83 ± 150.90	136.97 ± 90.39	558.88 ± 334.03^*∗∗∗∗*^
4	60.77 ± 49.94	264.03 ± 162.52^*∗∗∗∗*^	137.65 ± 104.61	287.49 ± 221.99^*∗∗∗∗*^
5	120.23 ± 74.62	448.04 ± 250.97^*∗∗∗∗*^	99.56 ± 80.81	440.18 ± 313.01^*∗∗∗∗*^
6	—	—	149.56 ± 105.60	328.61 ± 189.40^*∗∗∗∗*^

Average data are expressed as mean ± SD. ^*∗∗*^*p* < 0.01, ^*∗∗∗*^*p* < 0.001, and ^*∗∗∗∗*^*p* < 0.0001 versus the linear model.

## Data Availability

The data used to support the findings of this study are included within the article. Specific requests may be forwarded to the corresponding author.
